This article has been retracted.

# Effects of Sevoflurane versus Propofol on Endogenous Nitric Oxide Metabolism during Laparoscopic Surgery

**DOI:** 10.1155/2021/6691943

**Published:** 2021-02-03

**Authors:** Ning Wang, Jing Zhang, Ruiling Zhao, Bin Zhao, Yongzhang Li, Xiaoqing Zhang, Peng Liu

**Affiliations:** ^1^Department of Anesthesiology, Xinle Hospital, Shijiazhuang 050700, Hebei, China; ^2^Room of Operating, Xinle Hospital, Shijiazhuang 050700, Hebei, China; ^3^Department of Urology, Xinle Hospital, Shijiazhuang 050700, Hebei, China; ^4^Department of Urology, Hebei Hospital of Traditional Chinese Medicine, Shijiazhuang 050700, Hebei, China; ^5^Department of Anesthesiology, The Third Hospital of Hebei Medical University, Shijiazhuang 050051, Hebei, China

## Abstract

For laparoscopic surgery, it is very difficult to assess the effect of different medicines used in the surgical procedure on the surgical results. In the past, doctors could use sevoflurane to numb and calm patients. For decades, this type of treatment has been fairly reliable and effective, but for laparoscopic surgery, the use of sevoflurane can lead to a wide range of blood glucose changes, so in recent years, sevoflurane compared to propofol in laparoscopic surgery on endogenous and nitrogen oxide metabolism has been studied more and more. In this paper, a variety of research methods were used to study the phenomenon of shock and excessive anesthesia encountered by patients in the treatment process. Through observation and drug experiment of patients in different treatment courses and treatment stages, patients were asked to use sevoflurane and propofol to conduct double-blind experiments on their own drug effects. At the same time, through the long-term observation of patients with different diseases and patients who need laparoscopic surgery, the nitrogen oxide metabolism in patients with sevoflurane compared with propofol endogenous was studied and analyzed. Through three groups of different conditions, the experimental group, the blind test group, and the control group were studied. To conclude, in laparoscopic surgery, the use of sevoflurane compared with propofol can have a good impact on the endogenous drug and nitrogen oxide metabolism. It can achieve a good effect on the anesthesia effect of surgery, the maintenance of patient's physical signs and heart rate, which is very beneficial to the operation. *Conclusion*. Sevoflurane compared with propofol has a good effect on endogenous nitrogen oxide metabolism in laparoscopic surgery.

## 1. Introduction

In today's medical research, there are a variety of studies on the use of drugs in laparoscopic surgery to produce a good impact on the metabolism of nitric oxide in patients [1]. In a variety of studies, whether patients can achieve a stable state for their own signs during surgery is a problem that most doctors and researchers pay attention to. Due to the complexity of various factors in the operation, including the patient's psychological state, the patient's physical quality, and the doctor's status, in order to enable the doctor to have a stable working environment during the operation, whether the influence of sevoflurane compared with propofol on endogenous nitric oxide metabolism in laparoscopic surgery can achieve stable improvement has become a hot research area.

In recent years, a large number of foreign scholars have made excellent research on the effect of sevoflurane compared with propofol on endogenous nitric oxide metabolism in laparoscopic surgery. Bagia et al. used a large number of experimental research methods in its research, compared different patients in the experimental group and the control group using sevoflurane and propofol, and concluded that the use of this drug in laparoscopic surgery can greatly reduce the side effects of patients and improve the therapeutic effect [2, 3]. Chambers et al. used case comparison method to compare the drug use of different groups of patients in different course of disease. It was concluded that the curative effect of sevoflurane was slightly higher than that of propofol, but both drugs could play a very good effect [4]. In their study, Hida et al. used the case study method to study the adaptability of patients to the drugs in different course of disease when using the two drugs. It was concluded that the use of sevoflurane and propofol can well control the physical signs of patients in a good state [5].

A large number of scholars and researchers in China have done a lot of research studies on the efficacy of this drug in surgery. Takahashi et al. used a lot of literature research methods in their research. They studied the situation of patients who used sevoflurane and propofol during hospitalization and after discharge from hospital and concluded that patients using drugs can greatly reduce the burden of the body and improve the healing rate [6]. Kopman and Naguib used a lot of experimental comparison methods in their research and compared the patient's physical state and the healing process, and after a long-term study, it was concluded that the patient's physical signs discomfort was reduced a lot after using sevoflurane and propofol and achieved good therapeutic effect [7]. In their research, Wony et al. used experimental research method. They used a variety of drugs together with sevoflurane and propofol. Through experiments and observation, it was concluded that the research effect of sevoflurane was better than that of other drugs. It is an ideal drug [8].

In this paper, case study and experimental research were used to study different patients in control group, experimental group, and blind test group. At the same time, different pathological characteristics of patients, drug adaptation in various treatment processes, and specific effects of drugs on patients were studied and compared. In a large number of experiments and studies, the treatment of patients in the control group and the experimental group was studied and analyzed.

## 2. Effect of Sevoflurane versus Propofol on the Metabolism of Endogenous Nitric Oxide during Laparoscopic Surgery

### 2.1. Experimental Design of Endogenous Sevoflurane versus Propofol in Laparoscopic Surgery

#### 2.1.1. Experimental Design of Anesthesia Process

All the three groups were given general anesthesia without tracheal intubation. Oxygen (pure oxygen, 2 L/min) was given in the back of the operating room. After 2 min, propofol 1.5–2.5 mg/kg was pumped into group P at the rate of 300 ml/h, and 4–8 mg kg^−1^H^−1^ was maintained after patients' consciousness disappeared; etomidate was pumped 0.25–0.35 mg/kg at the same rate of 300 ml/h in group E, and etomidate was injected at a constant speed after patients' consciousness disappeared. In the EP group, etomidate 0.15 mg/kg was infused at the rate of 300 ml/h; then propofol 0.5–1.0 mg/kg was pumped at the same rate. After the consciousness disappeared, propofol was maintained at 4–8 mg kg^−1^H^−1^. If body movement occurs during the operation, which affects the operation, propofol 20–40 mg or etomidate 2–4 mg should be added. During the operation, if the patient has respiratory depression, the mandible was lifted and the mask was pressurized to give oxygen until the breathing recovers. If the mean arterial pressure is lower than 70 mmHg, it was corrected by intravenous injection of ephedrine 5 mg [9, 10]. If the heart rate is lower than 60 beats/min, intravenous atropine 0.25–0.5 mg is given to correct the problem. Patients with nausea and vomiting were treated with tropisetron hydrochloride 5 mg intravenously. Patients stopped infusion of propofol or etomidate at the end of the operation. The patients were infused with Ringer's lactate injection during the operation and were sent to the post-anesthesia recovery unit (PACU) for resuscitation. The patients were followed up on the first day after operation, including intraoperative awareness, injection pain, nausea and vomiting, and other adverse reactions [11, 12].

#### 2.1.2. Experimental Design of Operation

The types of gynecological operations by hysteroscopy include endometrial polypectomy, intrauterine adhesions decomposition, IUD removal, submucosal myomectomy, and mediastinal hysterectomy. After the surgeon disinfected and spread the towel, anesthesia induction was started, and the operation was started after the patient's consciousness disappeared. The irrigating fluid of hysteroscopy is mediocre isotonic fluid. The pressure of hysteroscopic dilatation was controlled at 80–120 mmHg. During the operation, the patient's condition was closely observed, and the occurrence of adverse events such as water poisoning and pulmonary embolism was on the alert [13–15].

The data were analyzed by SPSS17.0. The measurement data were expressed as mean ± standard deviation (*x* ± *s*). One-way ANOVA was used to compare the two groups. *t*-test was used for intragroup comparison. Chi-square test was used to compare the count data. Rank sum test was used to compare rank data. *P* < 0.05 means the difference is statistically significant [16, 17].

### 2.2. Experimental Design of Sevoflurane versus Propofol in Laparoscopic Surgery

#### 2.2.1. Experiment of Design Method

All patients were strictly prohibited from drinking and fasting before the operation. All patients were routinely given insulin one night before operation (daily dose range). They were stopped in the morning before operation. Blood glucose (mmol/L) was checked and recorded before operation. ECG, noninvasive blood pressure, pulse oxygen saturation (SpO_2_), bispectral index (BIS), and end expiratory carbon dioxide map were monitored after entering the operating room. All patients were given midazolam 2 mg 30 minutes before the operation. The blood glucose value was checked and recorded before operation, and then sodium lactate ringer injection was started. Etomidate (0.2 mg/kg iv), rocuronium (0.6 mg/kg iv), and sufentanil (0.5 UG/kg iv) were used for anesthesia induction, and laryngoscope tracheal intubation was used after administration [18, 19]. After anesthesia induction, low-dose glucose was infused at a rate of 0.05 g/kg/h, and the blood glucose values before anesthesia induction and after skin incision were recorded. Blood glucose was detected by blood glucose meter every 30 minutes after skin incision. The patients were randomly divided into two groups according to the data table. Propofol was infused at a rate of 5–10 mg/kg/h in the propofol group (group P), and 1.5–2.0 MAC (minimum effective alveolar concentration) was used in the sevoflurane group (group S) to maintain the depth of anesthesia, and the BIS value was maintained between 40 and 60 during the operation. At the same time, remifentanil was infused with micropump at the speed of 10–15 *μ*g/kg/h in both groups. At the end of the operation, neostigmine (0.04 mg/kg iv) and atropine (0.02 mg/kg iv) were used to reverse the residual neuromuscular block.

#### 2.2.2. Experimental Design of Observation and Detection

Heart rate (HR), blood pressure (NIBP), pulse oxygen saturation (SpO_2_), BIS, and end expiratory carbon dioxide (ETCO2) were recorded in both groups after entering the room and connecting the monitoring instrument. Blood samples were collected at each monitoring time point. Blood glucose values were measured immediately with blood glucose meter and blood glucose test paper. Blood glucose values (fbs0), before anesthesia induction (fbs1), at skin incision (fbs2), and 30 minutes, 60 minutes, and 90 minutes after operation (fbs3, fbs4, and fbs5), were recorded [20, 21].

#### 2.2.3. Statistical Design of Experiment

SPSS19.0 statistical software was used for data analysis. The measurement data were expressed by *X* ± *s* and were analyzed by *t-*test. The difference was statistically significant (*P* < 0.05).

### 2.3. Experimental Design of Sevoflurane versus Propofol on Endogenous Nitric Oxide Metabolism in Laparoscopic Surgery

After entering the room, the peripheral vein was opened and the radial artery catheterization was performed for dynamic pressure measurement. The standard monitoring items included electrocardiogram (ECG), pulse oxygen saturation (SpO_2_), end expiratory carbon dioxide (PetCO_2_), and bispectral index (BIS) [22, 23]. Both groups were given fentanyl 4 ug/kg, etomidate 0.2–0.4 mg/kg, and CIS atracurium 0.2 mg/kg for tracheal intubation, connected with a ventilator to control breathing, inhaled oxygen concentration 40%, volume control mode, tidal volume 8–10 ml/kg, frequency 12–15 times/min, end expiratory co230–40 mmhg, and fentanyl 1-2 ug/kg before skin incision. Continue to pump cisatracurium 0.1 mg/kg/h to maintain muscle relaxation before skin suture. Patients in the propofol group were given propofol TCI 2–4 ug/ml during operation, and patients in the sevoflurane group inhaled sevoflurane [24, 25].

#### 2.3.1. Design of Experimental Method

The sevoflurane vaporizer was closed and the fresh gas flow rate was increased to 6 L/min. BIS was used to monitor the depth of anesthesia and the concentration of propofol or sevoflurane was adjusted to maintain bis 40–60. In case of hypotension (systolic blood pressure < 90 mmHg or mean arterial pressure < 65 mmHg), ephedrine 10 mg was injected intravenously. If bradycardia occurred (HR < 60 beats/min), atropine 0.5 mg was injected intravenously. Ondansetron 8 mg was given routinely before the end of the operation to prevent postoperative nausea and vomiting. The operation time, fentanyl dosage, extubation time, and hemodynamic parameters were recorded. After the operation, the tracheal tube was removed and transferred to the post-anesthesia recovery unit (PACU).

After the operation, the patient-controlled intravenous analgesia (PCIA) was connected. The formula was fentanyl 0.02 mg/kg to 100 ml, the single dose was 2 ml, the background infusion volume was 0.5 ml/h, and the locking time was 5 minutes. The patients were observed with oxygen inhalation through nasal catheter in PACU for about 60 minutes. They were escorted back to the ward after they fully recovered, cough and swallowing reflex recovered, hemodynamic indexes were stable, and muscle strength recovered. Pain rescue treatment plan: if the patient requires or VAS score is greater than or equal to 7 points, flurbiprofen axetil (KAIFEN) 50 mg intravenous drip, if necessary, can be repeated within 24 hours, record the use of analgesic [26, 27].

#### 2.3.2. Design of Observation Experiment Index

The operation time, recovery time, fentanyl dosage, and hemodynamic changes of the two groups were compared, including blood pressure and heart rate before anesthesia, at the end of operation, after extubation, and after leaving PACU and returning to ward. The VAS scores (resting state and coughing) after extubation, PACU, 4 h, 12 h, 24 h, and 48 h after operation, and the cumulative dosage of fentanyl in the analgesia pump at 4 h, 24 h, and 48 h after operation were recorded. The number of PONV cases that occurred within 48 hours after operation, the number of pain relief drugs used, the length of hospital stay, the occurrence of possible adverse events (such as abdominal hemorrhage, reoperation, and incision infection), and the number of pain cases in 1 month and 3 months after discharge were also recorded [28, 29].

#### 2.3.3. Design of Statistical Methods

According to the previous clinical studies, the expected use of propofol compared with sevoflurane in the use of fentanyl has a 20% difference [30]. Based on the test level of 0.05 and assurance of 80% as the standard, 25 patients in each group are required. Therefore, 30 patients in each group are proposed to compensate for the cases that may fall off. SPSS19 statistical software was used for statistical analysis (IBM SPSS, Chicago, IL) [31]. Kolmogorov–Smirnov test was used to determine whether the data were of normal distribution. The measurement data were expressed as mean ± standard deviation (SD) and analyzed by independent sample *t*-test [32].

### 2.4. Experimental Design of Endogenous Propofol in Laparoscopic Surgery

The patient was intramuscularly injected with 0.1 g phenobarbital sodium before operation. General anesthesia began with intravenous induction anesthesia, fentanyl 2.5–4 *μ*g/kg, etomidate 0.2-0.3 mg/kg, and vecuronium 0.08–0.10 mg/kg. Endotracheal intubation was performed after muscle relaxation. The anesthesia machine was adjusted, the tidal volume of mechanical ventilation was set to 7–9 ml/kg, with respiratory rate of 10–12 times/min, and the end expiratory carbon dioxide partial pressure (PetCO_2_) was maintained at 35–40 mmHg. The patients were given propofol target-controlled infusion (TCI plasma target concentration 2–4 *μ*g/ml) (group A), sevoflurane inhalation 1%–3% (group B), propofol target controlled infusion combined with sevoflurane inhalation (group C), combined with vecuronium (used under muscle relaxation monitoring) and remifentanil (TCI plasma target concentration of 4 ng/ml) to maintain anesthesia.

ECG, heart rate, blood pressure, oxygen saturation, and other indicators were monitored by the monitor, and the blood pressure was maintained at ±15% of the basic value. Bispectral index was detected by depth of anesthesia monitor to keep BIS value between 38 and 45 [33]. The temperature of nasopharynx was maintained between 36.2°C and 37°C.

Vecuronium was stopped at 30 minutes after operation. Remifentanil and propofol were stopped before skin suture. Sevoflurane was stopped only after the drainage tube was placed, and the oxygen flow rate was increased to 5-6 L/min for lung flushing to accelerate its discharge.

After the operation, the patients were sent to the resuscitation room for natural recovery and extubation after recovery. The indication of extubation is as follows: be able to follow the instructions. They can open their eyes by themselves. The tidal volume is more than 5 ml/kg. The respiratory rate was between 15 and 24 breaths/min. Blood oxygen saturation was more than 95%. The time of eye opening and extubation was recorded. Sufentanil was given 1.5 *μ*g/kg D for intravenous analgesia. Blood pressure, heart rate, and oxygen saturation were monitored continuously within 7 days after operation to keep the patients in a stable and comfortable state within 7 days, so as to reduce pain and avoid upper respiratory tract infection.

#### 2.4.1. Experimental Design before Anesthesia

MMSE was used before anesthesia, 6 hours after operation, 24 hours after operation, 7 days after operation, 30 days after operation, and 6 months after operation. The patients and the doctors who scored were not clear about the group they belonged to. This score can assess the patient's attention, orientation, recall, calculation, language, and memory. POCD can be considered to have occurred when the score is less than 23, with the highest score of 30. 0–18 is severe cognitive impairment, 19–23 is moderate cognitive impairment, and 24–26 is mild cognitive impairment. MMSE score was used. MMSE is the most commonly used scale to examine cognitive function. Although the MMSE is simple and practical, different evaluators have different effects, which will produce a large deviation.

#### 2.4.2. The Experimental Objects and Methods of Operation

In this study, we followed the following principles:

1. Orientation: a total of 10 points: they are the day of the week; the date of the day; the month; what season; which year; where are we now: (province, city), (district or county), and (street or township); where's the place: the floor of the building, 1 point for each item, and 1 point for the day of the week.
2. Immediate memory: a total of 3 points, also known as initial memory or primary memory; it requires the examinee to immediately remember three objects with different properties. The name of the object should be continuous and clear, and not too fast. Repeat up to 3 times. Score according to the first answer, 1 point for each item. In addition, we should tell the examinees that the question will be asked later, so that the tested people are prepared.
3. Attention and computational power: a total of 5 points; for example, ask the examinee to reduce 7 continuously from 100. One point will be deducted for each mistake, which will be counted as 10 times, 0.5 point for each time. If there is a mistake in the middle, but the next answer is right, only one error is recorded. In order to avoid training effect, the arithmetic problem is given a different one each time.
4. Recall: a total of 3 points. The subjects were asked to name the three objects they were asked to memorize in advance, with 1 point for each item.
5. Language ability. ① Naming ability: a total of 2 points, show the examinee, watch and pen, and score 1 point for those who can say their names correctly. ② Language retelling ability: a total of 1 point; the test subjects are required to repeat a word of medium difficulty, but there is no rigid requirement on whether they use Putonghua or their intonation. ③ Level 3 command: a total of 3 points, handed to the subject, a piece of white paper. It is required to be tested. Hold this piece of paper with your right hand, and fold it in half with two hands. Because of this kind of operation, patients are usually in supine position in hospital, they can be placed on their stomach or chest (pay attention not to make secondary explanation, let alone demonstration action), 1 point for each of the three movements.

## 3. Comparison of Sevoflurane and Propofol on Endogenous Nitric Oxide Metabolism in Laparoscopic Surgery

### 3.1. Experimental Background

In today's laparoscopic surgery, most doctors use the traditional treatment, drug anesthesia and surgical treatment were performed on different patients. But this kind of treatment method, whether in the patient's adaptation degree or the patient's treatment effect, is not satisfactory. So sevoflurane versus propofol in laparoscopic surgery for endogenous treatment was invented.

### 3.2. Experimental Research Methods

#### 3.2.1. Experimental Research Method

The research method of this paper is to use the experimental research method, different patients in different control groups, drug treatment, nondrug treatment, and control treatment. After a long time of treatment and observation, patients can get real-time observation data for the adaptability of drugs.

#### 3.2.2. Case Study Method

In this paper, a case study method is used. Sevoflurane and propofol are used in several operations of patients, and then observation and interview are carried out in different signs of patients. The treatment results and experimental results are obtained from the feedback of patients.

#### 3.2.3. Literature Research Method

This paper uses the method of literature research to study and analyze a large number of clinical data of patients in the hospital, the feedback of patients in clinical treatment, and the real-time data of the hospital, so as to obtain a large number of research data.

### 3.3. Experimental Data Collection

In a large number of studies and experimental analysis, this paper obtained a large number of research data on the adaptability of patients to sevoflurane and propofol and the therapeutic effect of drugs. Get the patient's physical signs 30 minutes to 90 minutes before surgery, use sevoflurane and propofol to treat patients between 20–40 years old, and patients after use can improve the success rate of surgery by more than 8%.

## 4. To Compare the Effect of Propofol on Endogenous Nitric Oxide Metabolism in Laparoscopic Surgery

### 4.1. Experimental Analysis of Sevoflurane versus Propofol in Laparoscopic Surgery

The blood glucose of sevoflurane group at 30, 60, and 90 minutes after operation was significantly different from that before operation (*P* < 0.05); however, there was no significant change in blood glucose in the propofol group during operation (*P* > 0.05), as shown in Figure 1.

The stress response caused by perioperative surgery enhances the response of the neuroendocrine system, which leads to material metabolism disorder. The release of epinephrine, cortisol, and inflammatory mediators can lead to hyperglycemia, but even short-term hyperglycemia can also lead to the suppression of immunity of patients, thus increasing the risk of postoperative infection, resulting in delayed recovery, deterioration of the disease, and even death. But at the same time, proper and reasonable supplement of exogenous glucose can provide carbohydrate to decompose energy and reduce the decomposition of protein and fat during operation, which can not only prevent hypoglycemia and ketoacidosis during operation, but also facilitate wound healing after operation. Therefore, it is very important for the prognosis to choose the ideal anesthetic drugs and reasonable infusion of certain amount of glucose to keep the blood glucose fluctuation in a small range during the perioperative period.

### 4.2. Experimental Analysis of Propofol in Laparoscopic Surgery

The incidence of hypotension, respiratory depression, tongue base retroversion, and injection pain in groups E and EP was lower than that in group P (*P* < 0.05), but there was no significant difference between group E and group EP (*P* > 0.05); the incidence of PONV in groups P and EP was lower than that in group E (*P* < 0.05), and the incidence of PONV in groups P and EP was lower than that in group E (*P* < 0.05). There was no significant difference between the three groups (*P* > 0.05); there was no significant difference in bradycardia, myoclonus, and postoperative dysphoria among the three groups (*P* > 0.05); no intraoperative awareness occurred in the three groups, and the specific data are shown in Figure 2.

Propofol and etomidate are the two hypnotic intravenous anesthetics that are widely used in painless diagnosis and treatment. Propofol is a derivative of alkylphenol, which has high fat solubility and is not easily soluble in water. The anesthetic mechanism of propofol has not been fully elucidated. It is generally accepted that propofol binds to the *β*-subunit of GABAA receptor. Etomidate is an imidazole derivative, and the molecular mechanism of its anesthetic effect is not clear. Most people think that it is related to the regulation of GABAA receptor. Etomidate aqueous solution is unstable, and the incidence of pain at the injection site is high, which has been eliminated. Propofol and etomidate are both ultra-short-acting and powerful intravenous anesthetics, and they all take effect within one minute after administration. The results showed that the induction time of anesthesia in the propofol group was longer than that in the etomidate group, which may be related to the larger induction dose of propofol and the longer pump time. However, the induction time of etomidate combined with propofol was shorter than that of single anesthesia, and the induction dose was less, which indicated that the combined application of etomidate and propofol had synergistic effect and enhanced pharmacodynamics, which could shorten the induction time of anesthesia and reduce the dosage of each other.

### 4.3. Experimental Analysis of Endogenous Propofol in Laparoscopic Surgery

There was no significant difference in general condition and operation characteristics between the two groups. The heart rate of patients in the propofol group was slower than that in the sevoflurane group at the time of extubation, which may indicate that the cardiovascular response of propofol maintenance anesthesia patients after extubation is lighter and comfort is higher. The specific data are shown in Figure 3.

The VAS pain scores of patients in the propofol group after extubation, PACU, 4, 12, 24, and 48 hours after surgery and cough (*P* < 0.05, Figure 3) and the cumulative requirement of fentanyl at 24 hours after operation (364.4 ± 139.1 vs. 529.3 ± 237.9 *μ*g, *P*=0.002, Figure 4) were significantly lower than those in the sevoflurane group. There was no significant difference in nausea and vomiting within 48 hours after operation and pain at 1 month and 3 months after discharge between the two groups (*P* > 0.05). In addition, there were no significant differences in the frequency of postoperative pain relief, length of hospital stay, and adverse events between the two groups.

### 4.4. Experimental Analysis of Endogenous Nitric Oxide Metabolism in Laparoscopic Surgery

There were no significant differences in body weight, operation time, blood loss, infusion volume, education level, and intraoperative bispectral index (*F* = 1.67 – 2.05, *P* > 0.05).

In the same age group, the postoperative eye opening time and extubation time in group B were slightly longer than those in group A and group C, but the difference was not statistically significant (*F* = 0.10∼1.90, *P* > 0.05). In each group, with the increase of age, the time of eye opening and extubation gradually prolonged (*F* = 568.81∼728.63, *P* < 0.01).

### 4.5. Experimental Analysis on Endogenous Nitric Oxide Metabolism of Sevoflurane versus Propofol in Laparoscopic Surgery

There was no significant difference in average age, body mass index, operation stage, tumor grade, and muscle invasion between the two groups (*P* > 0.05). See Table 1 for details.

The results of intraoperative comparison between the two groups were as follows: (1) the average operation time of laparoscopic group was 168.15 ± 65.6 (min), and that of laparotomy group was 157.13 ± 63.05 (min) (*P*=0.429). (2) The difference of hemoglobin before and after operation: laparoscopic group: 8.97 ± 7.52 (g/L) and open group: 13.06 ± 11.07 (g/L) (*P*=0.044). (3) The average number of pelvic lymph nodes removed in the laparoscopic group was 21.83 ± 11.93, and that in the laparotomy group was 19.16 ± 10.24 (*P*=0.391). The average number of para-aortic lymph nodes removed in the laparoscopic group was 3.66 ± 2.23, and that in the open group was 2.66 ± 1.73 (*P*=0.387). (4) Intraoperative complications: in the laparoscopic group, blood transfusion occurred in 1 case, pneumothorax occurred in 1 case, no intraoperative complications occurred in the laparotomy group, and no intraoperative complications were recorded in other cases, because the number of cases was too small to be statistically compared.

## 5. Conclusions

In this paper, a large number of experimental research methods and case studies are used to study and analyze the efficacy of drugs in various situations. Sevoflurane and propofol can improve the success rate of surgery and promote the healing after surgery.

This paper studies the drug experiment of sevoflurane and propofol before operation. It is concluded that the patient can promote the operation process after taking the medicine. And it is concluded that sevoflurane as a new drug has a lot of help in the side effects of drugs, the effect of drugs, and the time of drug production. Compared with other drugs, the action time is shorter, the curative effect is strong, and the side effects are small.

Finally, through a large number of experimental researches and case studies, after a lot of treatment case studies, it is concluded that the use of sevoflurane and propofol in laparoscopic surgery is helpful for doctors to grasp the patient's physical signs, master the patient's treatment effect, reduce the patient's various accidents, and stabilize the patient's physical signs. Finally, after the experiment and research, it is concluded that the therapeutic effect of sevoflurane compared with propofol on endogenous nitric oxide metabolism in laparoscopic surgery is about 8% higher than that of propofol.

## Figures and Tables

**Figure 1:** Experimental map of propofol in laparoscopic surgery.

**Figure 2:** Experimental data of propofol in laparoscopy.

**Figure 3:** Effect of propofol on endogenous map in laparoscopic surgery.

**Figure 4:** Endogenous chart in laparoscopic surgery.

**Table 1:** Table of endogenous effects of propofol in laparoscopic surgery.

Sevoflurane	21.83 ± 11.93	19.16 ± 10.24	0.870	0.391
Propofol	3.66 ± 2.23	2.66 ± 1.73	0.915	0.387
Blood transfusion	1	0		
Pneumothorax	1	0		
Injury caused by puncture	0	0		
Air embolism	0	0		

## Data Availability

No data were used to support this study.
